# Construction of Mental Health Knowledge Service Model Based on Online Medical Community

**DOI:** 10.1155/2022/1907074

**Published:** 2022-06-30

**Authors:** Jingxiu Xu, Xueguang Li, Xianju Wang, Bifeng Li, Zhihua Hu, Feng Wang, Xiaoyan Liu

**Affiliations:** ^1^School of Computer Science and Technology, Huanggang Normal University, Huanggang 438000, Hubei, China; ^2^China Research Institute of Radiowave Propagation, Xinxiang 453000, Henan, China; ^3^School of Physics and Electronic Engineering, Fuyang Normal University, Fuyang 236037, Shenyang, China; ^4^Jike ICT Support Department, Zhejiang Wasu Broadcast & Network Co., Ltd., Hangzhou 310000, Zhejiang, China; ^5^Department of Virtual Reality, Jiangxi Tellhow Animation Vocational College, Nanchang 330200, Jiangxi, China

## Abstract

This paper discusses a common mental disorder prevention mode to improve residents' mental health quality and achieve the “comprehensive and fine-grained” mental health education knowledge service. The construction of mental health knowledge service model is conducive to accurately grasp the group cognition and psychological changes and take the initiative to make decisions. This paper analyzes the needs of mental health education knowledge service system and combs the research status of applying information technology and artificial intelligence to mental health education at home and abroad, the resource data of five major online medical communities at home and abroad were screened and mined, and the mental health feature tags of college students were extracted. Based on the existing mental health diagnosis experience database and multisource text, reuse and optimize ontology integration method to systematically construct mental health education ontology. Taking mental illness as an example, the rule base is constructed and the personalized recommendation service of mental health is realized. The service model can infer and output all kinds of diagnosis and treatment knowledge to provide users with intelligent mental health education knowledge services.

## 1. Introduction

The “national mental health law of People's Republic of China” issued by NPC Standing Committee points out that the relevant departments at or above the county level should take measures to strengthen mental health and prevent mental disorders, so as to improve the level of public mental health. “The national mental health work plan (2015–2020)” issued by the National Health and Family Planning Commission of the PRC points out that we should actively pay attention to the psychological and behavioral problems of women, children, the elderly, and occupational groups and provide public welfare services for mental health to the public. “The New Generation of Artificial Intelligence Development Plan” issued by the State Council of the PRC proposes the fact that artificial intelligence technology will be used for early warning of group psychological changes and active decision-making response.

Zhong Nanshan, a famous respiratory expert in China, said the following: half of health is mental health, and half of disease is mental disease. The knowledge of mental health education enables patients to understand the pathological knowledge, reasonably use the methods of elimination and counseling for disease management, promote patients' self-management and disease rehabilitation, and at the same time enable the mental health groups to establish scientific health awareness in advance. Experts and scholars have carried out a lot of research in this area. Wang combed the evolution and development course of college students' mental health education policy [1]; Wang et al. obtained the enlightenment of relieving network health anxiety by extracting network health anxiety factors [2]; Li et al. put forward the reform direction of mental health education system in the new period of network and constructed specialized mental health education platform [3, 4]; Peng analyzes the mental health education of college students by using systematic guiding ideology in the aspects of integrity, hierarchy, and purpose [5]. Yang et al. used, based on the user information needs theory modeling, the questionnaire analysis to obtain the college students mental health information conscious needs of five trigger path conclusions [6].

At present, the research methods of user mental health knowledge service are mostly theoretical analysis. Some scholars have designed questionnaires to evaluate mental health and analyze the results, and others have drawn conclusions through bibliometric analysis [7], ignoring the importance of mining a large number of valuable text data amounts in online medical community. With the advent of the era of artificial intelligence, personalized and intelligent service of users' mental health knowledge is scarce, which cannot meet the real needs of users searching for diversified and professional psychological knowledge in the new era. The innovation of this paper is based on the theory of knowledge engineering, which realizes the research of online medical community mental health education knowledge base construction and intelligent service. The main online medical community resource data at home and abroad are screened and mined to extract mental health feature tags. Based on the knowledge map of traditional Chinese medicine, the existing experience base of traditional Chinese medicine knowledge service platform, and multisource text, the ontology knowledge base of mental health education is systematically constructed by using ontology integration method, and the ontology rule base is constructed by taking mental diseases as an example. The platform of mental health guidance and mental disease prevention and control knowledge service was developed to provide intelligent mental health education knowledge service for users.

## 2. Related Research

### 2.1. Online Medical Community Analysis

At present, most areas at home and abroad have achieved network coverage, it is convenient for patients to acquire mental health education knowledge, and the domestic online medical community mainly has “https://www.xywy.com,” “https://www.39.net,” “https://www.haodf.com,” and “https://www.chunyuyisheng.com.” “https://www.xywy.com” has launched a psychological channel to popularize the knowledge of heart disease cases, heart medicine introduction, psychological common sense, mental health care, and psychotherapy and can do simple psychological tests. “https://www.39.net” has launched a psychological channel to popularize information such as psychological information, mental health care, psychological feelings, psychological encyclopedia, psychological services, and special planning.” “https://www.haodf.com” and “https://www.chunyuyisheng.com” launched the psychiatry online expert consultation service; the foreign online medical community “Medscape” launched the psychiatry online expert consultation service. The information resources provided by these online medical communities not only popularize the knowledge of mental health, but also have several shortcomings: ① due to the different mental health status of each user, they cannot meet the needs of individual mental health consulting services; ② most communities did not set up personalized Q &and A board and feedback communication board; ③ online expert consultation is a charge item, and there is no free consultation service; ④ the condition and treatment information of purchased online expert consultation users is not transparent, and other users cannot refer to the information of mental illness cases.

### 2.2. Online Mental Disease Search

Depression, anxiety disorder, sleep disorder, and mania are the most common forms of many mental illness. Using “depression,” “anxiety disorder,” “sleep disorder,” and “mania” as keywords, the overall daily average of Baidu search index for these four common mental illness in the past four years (2016 to 2020) is shown in Table 1 and Figure 1; there is a steady upward trend in people's attention to mental illness. These indicators reflect the use of search engines to obtain a large amount of mental health counseling related knowledge; there is a large demand for mental illness symptoms and manifestations, treatment, and other knowledge.

To sum up, it is convenient to use Internet search engine tools to find keywords, but at the same time there are many unwanted advertising promotion links and useless links, which cannot provide personalized intelligent services. Users' access to psychological counseling knowledge is very limited, and the mental health education is fragmented, and the pertinence is not strong, which cannot meet the needs of intelligent knowledge services.

### 2.3. Construction of Ontology Knowledge Base Theory

The function of ontology is to build domain model. The construction of ontology knowledge base can solve heterogeneous data sharing, knowledge sharing, knowledge reuse, and system integration. Tang et al. constructed the ontology knowledge base of chronic disease health education and realized the automatic question and answer of health knowledge and individualized recommendation of health care plan [8]; Cui, combined with expert knowledge, taking psoriasis as an example, constructed the ontology knowledge base of TCM diagnosis and treatment [9]; Zhai et al. constructed the related knowledge map by studying the keywords of CNKI literature [10]; Li et al. used ontology knowledge base construction method to build ontology modeling and rule base, knowledge map visualization research [11–13]. Through the semantic analysis of Unified Medical Language System (UMLS) and Traditional Chinese Medicine Language System (TCMLS), Xu et al. realized the transformation of STKOS to RDF, which provided the basis of medical concept research of mental health specialty [14–17]; Chen et al. used multiple logic regression method to analyze the mental health status of Chinese doctors working in intensive care unit [18].

### 2.4. Intelligent Service Model

The establishment of intelligent service model can provide knowledge service and decision-making intelligent service conveniently. Through open decoding, spindle decoding, and selective decoding, Xu et al. concluded the types of health information needs of the elderly and constructed a community-based cooperative health information service model for the elderly [19]. Xiong et al. build the knowledge base of chronic disease ontology and develop the service platform of chronic disease knowledge by collecting the data of chronic disease resources, literature, and expert knowledge online [20]. Based on knowledge engineering research methods, Tang et al. constructed a prototype system of enterprise bankruptcy prediction and effectively carried out enterprise bankruptcy prediction [21]; Gan et al. constructed the intelligent medical diagnosis system mechanism based on Jess fuzzy reasoning and provided the idea of intelligent resource sharing [22]. Li et al. combed the research and elements of information retrieval system and digital library and expounded the elements of knowledge service platform evaluation [23]. Wang constructed a user-centered intellectual property information service system model framework by designing questionnaires and interviews [24]; Phoebe Barnett et al. used the system retrieval and meta-analysis to construct the college students' psychological disorder intervention and prevention system [25, 26]. Aiming at the problems in the mental health education of college students, Kaixin Gong constructs a theoretical model of the key extensible strategies of mental health education for college students [27, 28].

To sum up, a small number of literatures at home and abroad use text data mining, machine learning, Internet of things technology, and knowledge mapping to build mental health ontology knowledge base. Personalized recommendation system has basic theoretical research, but there are few researches on the construction of mental health knowledge service model based on online medical community. The main problems are as follows: first, the research object is too wide, lacking systematic construction of mental health education ontology knowledge base for users; second, the research methods of mental health education intelligent service model are mostly theoretical model research; third, there is lack of organic integration of the two research and better service personalized knowledge is needed.

## 3. Knowledge Service System Model of Mental Health Education

Mental health education knowledge base and intelligent service system aim to provide online intelligent and personalized mental health education knowledge service for users. In this paper, the online medical community resources as the main data source, based on the ontology knowledge engineering construction theory, build mental health knowledge service model based on online medical community. The construction idea of this model is mainly based on the characteristics of good operation performance, practicability, and intelligence of the system, as shown in Figure 2. The framework mainly includes data acquisition module, knowledge base construction module, and knowledge service module. The data acquisition module provides all kinds of data resources needed by the knowledge base, which is the physical basis of mental health education knowledge service. The core part of this study is the knowledge base construction module, which effectively organizes all kinds of knowledge resources and systematically constructs mental health ontology knowledge base through ontology integration. Knowledge service module is the part of user interface. Personalized recommendation service is the key part of intelligent service.

### 3.1. Data Acquisition Module

This study is mainly oriented to multisource data, which needs feature analysis and mental health label extraction through keyword statistics. Data collection sources are five main online mental health medical communities at home and abroad, core documents of mental health medicine, electronic medical records, monographs, psychological test reports, interview records, information resources of college students, expert knowledge base, hospital information system (HIS), and so on.

The online mental health care community mainly has “https://www.xywy.com,” “https://www.39.net,” “https://www.haodf.com,” and “https://www.chunyuyisheng.com.” These online medical communities have special psychological channels or psychopharmacology; psychological channels or psychopharmacology data format is basically text data, obtained through crawler collection of psychiatric labels; each mental illness has expert doctor Q & A symptoms, medication, diet therapy, health care and personal advice, and other knowledge. Delete the text similar or repeated content and finally extract 1739 data as sample data stored. Part of the sample data collection results is shown in Table 2.

The core literature of mental health medicine at home and abroad refers to the Chinese core literature, foreign core literature, monographs, and so on related to mental diseases. We can access the literature related to mental diseases or mental health knowledge at home and abroad through python. The mental health clinical information system records the basic information of patients, family history, and psychological test reports. The psychological test report refers to the mental health records that are established by doctors according to the test results after each psychological patient arranges the online psychological test in the hospital. These data can be obtained through the integrated access of database connection interface, and the paper data can be obtained through manual data processing.

Expert knowledge base refers to the accumulation of professional knowledge and treatment experience of experts in mental health field for many years, clinical drug use knowledge, clinical experimental examination and medical literature organized by senior medical editors, etc., stored in expert system. Hospital information system (HIS) is a valuable information platform for authorized users by using electronic computer and communication equipment to provide patient diagnosis and treatment information for all departments affiliated to the hospital. It provides patient diagnosis and treatment information and medical record management subsystem medical record and electronic medical record. These management information system data can be obtained through database connection interface integration access.

### 3.2. Mental Health Education Knowledge Base Module

Mental health education knowledge resource database is constructed by multiple data sources; the data should be cleaned because of the redundancy of all kinds of online mental health medical resources, literature, and other text information. Most of the collected data are semistructured text data or unstructured data. Because the form of data structure is not uniform, it needs to be regulated, converted, and integrated. Natural language processing and knowledge extraction are used to construct ontology knowledge base. Finally, the ontology knowledge base is generated by transforming the existing empirical ontology library, multisource text subject word collection, and statute to the concept, instance, relation, attribute, type, and constraint.

#### 3.2.1. Text Analysis and Natural Language Processing

The purpose of text analysis mining is to mine the characteristics of mental health knowledge in a large number of potentially useful text data. The text analysis and mining tool adopts the nlpir-ictclas Chinese word segmentation system of Professor Huaping Zhang, at Chinese Academy of Sciences. The extracted knowledge can be referred to the data table PSY which is the source of supersaurus MEDEF and the language system of Traditional Chinese Medicine Language System (TCMLS), which is a large computerized language system based on the subject system of traditional Chinese medicine. It contains about 100000 concepts, 300000 terms, and 1.27 million semantic relationships.

In order to calculate the mental health knowledge feature tag, this study specifies TF-IDF to classify the cleaned document *d*, and the word frequency (TF) counts the frequency of a mental health knowledge tag in document *d*. Here, *n* represents the number of documents classified and *t* represents the label words appearing in document *d*. For the word *t*_*i*_ in a specific document, its importance can be expressed as the following formula:

(1) $$\begin{array}{c} tf_{i,j}=\frac{n_{i,j}}{\sum_{k}n_{k,j}}, \end{array}$$

where *n*_*i*,*j*_ is the word *t*_*i*_ in document *d*_*j*_. For the number of occurrences in *j*, TF-IDF assumes that the high frequency has a high weight, while the inverse document frequency (IDF) is inversely proportional to the word frequency (TF), which is a measure of the general importance of a word. Its formula is as follows:

(2) $$\begin{array}{c} {\text{IDF}}_{i,j}=\text{log}\left(\frac{D}{1+j}\right). \end{array}$$

After obtaining TF and IDF values, then multiply them to obtain TF-IDF values. The formula is as follows:

(3) $$\begin{array}{c} \text{TF}{\text{.IDF}}_{i,j}={\text{TF}}_{i,j}*{\text{IDF}}_{i,j}. \end{array}$$

Text analysis and knowledge extraction in this study are mainly divided into three stages: artificial primary selection, text preprocessing, and word frequency TF-IDF feature extraction. (1) In the aspect of artificial primary selection, the collected online psychotherapy community sample data are artificially screened to delete the information independent of the subject text. (2) As for text preprocessing, Python stuttering word segmentation system is used to preprocess the characteristics of natural language, to establish a stop using words database and mental health dictionary, and to remove the common stop words with little meaning. (3) With regard to word frequency TF-IDF feature extraction, online mental health community data, and related scientific and technological documents, electronic reports and other materials from artificial primaries are used as sample corpora, four common medical terms for mental illness are added to the corpus, and the weight factor is used for feature extraction, and then TF-IDF feature extraction algorithm is used. The main purpose of TF-IDF feature extraction algorithm is to optimize the segmentation effect and improve the accuracy of keyword extraction and text mining. Main mental health knowledge label word frequency TF-IDF feature extraction results are shown in Table 3.

#### 3.2.2. Construction of Ontology Knowledge Base

Ontology is generally called domain model or conceptual model, which is a theory about the existence of some relationship among various objects, object attributes, and objects in a specific knowledge field. Ontology knowledge base is a concrete application based on ontology model construction; the general ontology knowledge base construction adopts manual, automatic, or semiautomatic methods. The user mental health education knowledge base consists of the existing experience knowledge base and the mental health ontology knowledge base. Experience knowledge base needs to select HIS, knowledge service platform of traditional Chinese medicine, and other multisource heterogeneous text subject word knowledge from existing knowledge base, listening to the advice of medical psychological experts and determining the scope of mental health ontology knowledge and standardized processing.

Combined with the feature extraction of mental health tag TF-IDF in Table 3, based on the existing empirical knowledge base and multisource heterogeneous text keywords, the ontology knowledge base is systematically constructed through ontology integration [28]. The important terms and concepts in mental health education ontology are extracted, and the framework of mental health education ontology is established. This paper defines classes and their levels, attributes, and attribute types, as well as values, semantic relations, and constraints and constructs ontology knowledge base with high practical value according to the actual needs of users' mental health. Ontology knowledge base building tools can be used by Resource Description Framework (RDF), Resource Description Framework Schema (RDFS), Web Ontology Language (OWL), Protégé, etc.; the inference tool Jena, Jess is a rule-based inference machine subsystem for retrieval of process inference to obtain high-performance mental health knowledge. Through the learning of this knowledge, users can achieve mental health self-management, effective prevention, and control of mental diseases and diagnosis.

### 3.3. Knowledge Server Module

The construction of this module is based on the effective organization of ontology knowledge base, which changes the single mental health education mode in the past and transforms into the knowledge service form of mental health education at many levels of vision. Using the advantage of resource utilization and software architecture technology in the network age, the intelligent service prototype system of mental health education is constructed, which is convenient for users to have a good service interface to acquire knowledge. This prototype system mainly constructs online psychological testing service, mental health education service, psychological question and answer personalized recommendation service, mental health prevention intervention service, and psychological dictionary service.

#### 3.3.1. Online Psychological Testing Services

In view of the needs of users' self-control of psychological diseases, online psychological tests are arranged regularly, and the test results can be used as reference. At the same time, in order to protect the personal privacy of users, the prototype system of anonymous login service for users carries out online psychological testing and generates a psychological test analysis report with reference significance and returns it to the users to meet the needs of users' convenient and visual access to their own health index testing services.

#### 3.3.2. Mental Health Education and Mental Health Preventive and Intervention Services

Mental health education services through the introduction of the current mainstream knowledge of mental illness popularize users psychological encyclopedia knowledge, such as the etiology of these illnesses, health therapy, drug treatment, and prevention mechanisms. Mental health prevention and intervention service provides professional and systematic treatment knowledge, reasonable exercise knowledge, extensive interest and hobby knowledge, physiotherapy knowledge, self-stress knowledge and diet knowledge, and other knowledge services to meet the needs of users' self-psychological health education management.

#### 3.3.3. Psychological Q & A Personalized Recommendation and Psychological Dictionary Service

The traditional online medical community simply achieves simple keyword link matching. Psychological Q & A personalized recommendation is based on the ontology knowledge base of patient and psychological expert question and answer for query and retrieval [29, 30], and using Protégé-OWL Extension Tool Semantic Web Rule Language SWRL Reasoning Rules provides psychological illness guidance and personalized knowledge services. It can recommend the prevention and treatment of mental illness and meet the needs of individualized guidance of mental health. The psychological dictionary service displays the existing mental health professional vocabulary and the new psychological hot words and annotates and explains them, so that uses can explore the mental health knowledge and new trends.

## 4. Construction and Reasoning of Ontology Knowledge Base of Mental Health Education

In order to meet the needs of users' mental health education knowledge service, this paper practices the optimized knowledge base of mental health education ontology and takes mental illness as the carrier to realize the connection and sharing of mental health education knowledge base and mental illness knowledge. Based on the tool Protégé，developed by Stanford University, this paper constructs the ontology knowledge base of mental health education by seven-step manual method, using semantic web rule language OWL to describe knowledge, to meet the needs of reasoner inference machine, to establish reasoning based on mental illness ontology and reasoning based on mental health rules, and to complete the triple mapping mechanism of OWL to RDF. It realizes the need of individualized recommendation service for users' mental health. Based on the ontology knowledge base of mental health education and the rule base of mental illness, the prototype system of intelligent service for mental health education is constructed.

### 4.1. Construction of Ontology Database of Mental Health Education

#### 4.1.1. Definition and Hierarchy of Classes

OWL ontology construction of mental health education knowledge service is mainly composed of class, subclass, object attribute, data attribute, instance, and a series of rules. The ontology of mental health education includes six important superclasses, which are used to describe abstract entity objects, namely, self-management of mental patients, mental experts, mental diseases, prevention of mental diseases, mental dictionaries, and psychological Q & A. The concept map of mental health education ontology is shown in Figure 3, and the concept map of mental diseases ontology is shown in Figure 4. Subclasses inherit the abstract characteristics of the parent class and represent a smaller range of entity concepts. The construction of the whole class is organized in a hierarchical structure. After defining all superclasses, classes, and subclasses and running the visualization tool Onto Graf, the mental health knowledge service ontology is shown in Figure 5.

#### 4.1.2. Property Definitions

After the ontology and class of mental health education are defined, the attribute of each class needs to be defined. The principle of attribute definition is to define according to the actual needs of domain class. Attributes mainly include object attributes and data attributes. During building, you need to define attribute name, definition field, and value field. The definition of some data attributes of mental illness ontology library is shown in Table 4, and the definition of some object attributes of mental illness ontology library is shown in Table 5.

### 4.2. Construction and Reasoning of Mental Health Education Rule Base

The construction of rule-based reasoning database in this paper is based on TCM knowledge map, TCM knowledge service platform, and online medical community resources. To improve the quality of personalized recommendation service for mental health, we need to extract the accumulated experience of psychological experts related to this study, such as medication and selection of psychiatrists and diet, and establish a rule base. Use Protégé-OWL Extension Tool Semantic Web Rule Language SWRL Reasoning Rules, in order to use the standard language of semantic web directly; format conversion is not carried out; SWRL is represented based on RDF; that is, OWL and RDF improve semantic reasoning. Use drools rule engine to realize rule knowledge reasoning of mental health education ontology knowledge base. The process of SWRL rule editing and reasoning is shown in Figure 6. Some rules of mental illness are extracted as follows:

1. Rule 1: depression patients eat caffeine carefully.
2. Rule 2: depression patients eat less high-sugar food.
3. Rule 3: patients with anxiety disorder eat caffeine carefully.
4. Rule 4: depression patients are suitable for spa recuperation.
5. Rule 5: insomnia patients can take Bailemian capsule for treatment.

### 4.3. Prototype of Mental Health Knowledge Service System

In order to meet the needs of users to obtain mental health education knowledge service, the author developed a mental health knowledge service prototype system based on ontology and semantic network. The development environment of the system is JAVA, the development version adopts JDK 1.8, the IDE development tool adopts Eclipse, the server adopts Tomcat 7.0, the database adopts MySQL, and the main interface of the mental health knowledge service prototype system is shown in Figure 7.

By using the mental health knowledge service prototype system, users can log in to realize anonymous online psychological test and know their mental health in time. According to the reference opinions of the test results, such as depression, you can enter depression in the text box and click to find it, which will display the condition introduction, online doctor recommendation, drug recommendation, and health recommendation of depression, so as to realize the personalized and convenient service of further seeking medicine. According to the experts recommended by the system, we can consult experts online or find specialized psychological medical institutions offline to achieve more professional diagnosis and treatment. For mental health users, you can click to find common mental health education knowledge and mental health prevention and intervention knowledge, consult the psychological dictionary, and do well in mental disease prevention in advance. The prototype system is helpful for users to realize self-management of mental health education effectively.

## 5. Conclusion

Mental health knowledge service plays a very important role in the self-prevention and control of mental diseases, and it is also one of the hot spots in the field of mental health and mental disorders. In view of the shortcomings of the research status in this field, this paper uses text data mining method to screen and mine the main online medical community resources, extract the user mental health feature tags, and systematically construct the mental health knowledge service ontology knowledge base based on the traditional Chinese medicine knowledge map, the existing experience base of the traditional Chinese medicine knowledge service platform and multisource text. Taking mental illness as an example, the ontology rule base is constructed, and the prototype of mental health knowledge service system is developed. This knowledge base realizes the integration and sharing of multisource data such as mental health knowledge, drugs, and experts. This study is conducive to accurately grasp the user's psychological changes and take the initiative to make decision response and has practical significance for the majority of users' self-prevention and control of mental diseases and self-education management.

The future research needs to improve in the following aspects: research the automatic construction technology of ontology knowledge base, realize the automatic construction of ontology, and improve the efficiency of building ontology knowledge base of mental health education knowledge service to achieve more accurate and detailed requirements of personalized reasoning rule base creation. Through the user experience to continuously improve the mental health knowledge service system upgrade needs, these will be the direction of future research efforts.

## Figures and Tables

**Figure 1:** “Four types of common mental illness” Baidu search index in the past four years average daily.

**Figure 2:** The model construction of mental health education knowledge service system.

**Figure 3:** Concept map of mental health education ontology.

**Figure 4:** Concept map of mental illness ontology.

**Figure 5:** Mental health knowledge service ontology.

**Figure 6:** SWRL rules editing and reasoning process.

**Figure 7:** Mental health knowledge service prototype system.

**Table 1:** Four types of common mental illness and related keywords and Baidu search index daily average in recent four years.

Mental illness	Related keywords and Baidu index

Depression	Symptoms and manifestations of depression, 1671; depression treatment, 474; what to eat for depression, 44
Hypnosis	Symptoms and manifestations of insomnia, 139; insomnia treatment, 316; what to eat for depression, 320
Anxiety disorder	Symptoms and manifestations of anxiety, 1941; treatment of anxiety disorders, 151
Schizophrenia	Symptoms and manifestations of schizophrenia, 226; schizophrenia treatment, 107

**Table 2:** Results of online mental health expert consultation.

Type of illness	Sequence	Content
Depression	1	Watch out! The longer the time you play with your phone, the higher the risk of depression!
	2	Depression may be around you. Be careful with these symptoms
	3	Changing your diet may relieve depression
	…	
	532	Depression will become the primary cause of disability! Study: socializing more prevents depression

A hypnosis	1	Wake up until 3.4 a.m. What should I do?
	2	How to distinguish between bad sleeping habits and sleep disorders?
	3	How does insomnia do? Eating more of these foods will help you sleep comfortably
	…	
	450	Etiology and treatment of insomnia

Anxiety disorder	1	Can TCM treat anxiety and insomnia?
	2	Anxiety headache, how to relax?
	3	Can anxiety disorder cause persistent dizziness tinnitus?
	…	
	412	Guidelines for comprehensive treatment of anxiety disorders

Schizophrenia	1	Watch out! Loss of appetite may be caused by schizophrenia...
	2	Schizophrenia patients with insomnia should be sure to guard against suicide risk
	3	Can schizophrenia recover?
	…	
	345	What is good to eat for schizophrenia?

**Table 3:** Main mental health knowledge label of feature extraction TF-IDF.

Feature word	Frequency	TF-IDF
Depression	99	0.464
Treatment	51	0.432
A hypnosis	42	0.337
College students	39	0161
Depression	32	0.155
Emotions	30	0.218
Psychological	27	0.224
Anxiety	23	0.203
Patients	21	0.158
Sleep	18	0,168
TCM	12	0168
Hospital	15	0.102
Life	12	0.167
Relax	13	0.168

**Table 4:** Some data attributes of mental illness ontology database.

Data attribute	Domain	Range

Attending physician	Psychological specialists	xsd:string
Patient's name	Psychiatric patients	xsd:string
Age of patients	Psychiatric patients	xsd:int
The sex of the patient	Psychiatric patients	xsd:string
Food	Psychiatric patients	xsd:string

**Table 5:** Some object attributes of mental illness ontology database.

Object properties	Domain	Range

Treatment	Psychological specialists	Insomnia/anxiety/depression
Cautious food	Psychiatric patients	Diet
Less food	Psychiatric patients	Diet
Convalescent	Psychiatric patients	Health maintenance
Take medicine	Psychiatric patients	Medicine

## Data Availability

The data used to support the findings of this study are available from the corresponding author upon request.
